# Novel insights into *Pinus* species plastids genome through phylogenetic relationships and repeat sequence analysis

**DOI:** 10.1371/journal.pone.0262040

**Published:** 2022-01-19

**Authors:** Umar Zeb, Xiukang Wang, Sajid Fiaz, Azizullah Azizullah, Asad Ali Shah, Sajjad Ali, Fazli Rahim, Hafiz Ullah, Umed Ali Leghari, Weiqiang Wang, Taufiq Nawaz

**Affiliations:** 1 Department of Biology, The University of Haripur, Khyber Pakhtunkhwa, Pakistan; 2 College of Life Sciences, Yan’an University, Yan’an, Shaanxi, China; 3 Department of Plant Breeding and Genetics, The University of Haripur, Haripur, Pakistan; 4 Department of Bioinformatics and Biotechnology, Government College University Faisalabad, Faisalabad, Pakistan; 5 Department of Botany, Bacha Khan University Charsadda, Khyber Pakhtunkhwa, Pakistan; 6 Departement of Botany, University of Chitral, Khyber Pakhtunkhwa, Pakistan; 7 Department of Agriculture, Mir Chakar Khan Rind University, Sibi, Balochistan, Pakistan; 8 Department of Food Science and Technology, The University of Agriculture Peshawar, Khyber Pakhtunkhwa, Pakistan; Anhui Agricultural University, CHINA

## Abstract

*Pinus* is one of the most economical and ecological important conifers, model specie for studying sequence divergence and molecular phylogeney of gymnosperms. The less availability of information for genome resources enable researchers to conduct evolutionary studies of *Pinus* species. To improve understanding, we firstly reported, previously released chloroplast genome of 72 *Pinus* species, the sequence variations, phylogenetic relationships and genome divergence among *Pinus* species. The results displayed 7 divergent hotspot regions (*trnD-GUC*, *trnY-GUA*, *trnH-GUG*, *ycf1*, *trnL-CAA*, *trnK-UUU* and *trnV-GAC*) in studied *Pinus* species, which holds potential to utilized as molecular genetic markers for future phylogenetic studies in *Pinnus* species. In addition, 3 types of repeats (tandem, palindromic and dispersed) were also studied in *Pinus* species under investigation. The outcome showed *P*. *nelsonii* had the highest, 76 numbers of repeats, while *P*. *sabiniana* had the lowest, 13 13 numbers of repeats. It was also observed, constructed phylogenetic tree displayed division into two significant diverged clades: single needle (soft pine) and double-needle (hard pine). Theoutcome of present investigation, based on the whole chloroplast genomes provided novel insights into the molecular based phylogeny of the genus *Pinus* which holds potential for its utilization in future studies focusing genetic diversity in *Pinnus* species.

## Introduction

*Pinus L*. (Pinaceae) is an important genus of conifers with more than 230 species. It is a broadly distributed in temperate zones of Northern Hemisphere [1]. Pines include important tree species which are commercially used in pharmacology and wood pulp industries around the world. Genus *Pinus* is divided into two subgenera *Strobus*, (Haploxylon) and *Pinus* (Diploxylon) [2]. Moreover, anatomical, molecular, and morphological evidence strongly reinforced divergence of *Strobus* and *Pinus*, respectively [3]. Because of ecological importance and diversity, genus *Pinus* prove a best model for molecular study of conifers. *Pinnus* genomes are extremely large (c. 20–40 Gb) and shown no evidence of recent polyploidy or chromosomal duplication. Pine chromosomes (2n = 24) are uniform both in number and appearance, owing to lack of major distinguishing physical features [4].

The phylogenetic tree displayed evolutionary relationships among different biological species based on similarities and differences for their maternal characteristics. Moreover, phylogenetic relationships in *Pinus* species are regularly studied through genome sequencing [5]. The whole chloroplast genome has numerous features e.g., small in size, conserved structure, maternal inheritance, and species identification is broadly applied for evolutionary studies [6]. Recently, an extremely divergent region in plant plastome has been identified called "hotspot region" and served an useful genetic marker for phylogeny and evolutionary studies of genus *Pinus* [7]. Previous studies showed that the genus *Pinus* had shared several genomic sequence variations for cp DNAs owing to their recent divergence radiation, regular interspecific and introgression gene flow among species [8]. The low degree of genomic divergence among *Pinus* species has been attributed to a large number of molecular evolution takeing place in related species [9]. Therefore, it hold integral importance to understand complete phylogenetic relationships of *Pinus* species to understand the underlying genetic mechanisms controlling its diverse features [10].

Complete chloroplast genome are circular DNA molecules, had a quadripartite shape with large single copy (LSC) region, a small single copy (SSC) region, and two inverted repeats (IRs) regions [6]. Previous studies had revealed that plastid DNA of gymnosperm plants were extremely maintained in genome structure, order and gene contents [11]. The repeat sequence analysis in plastome contributes to various cellular functions including RNA editing, gene mobility and gene evolution [12]. Repetitive sequences are categorized into three modules: local repeats (simple sequence repeats (SSRs) and tandem repeats), families of dispersed repeats (mostly transposable elements and retro-transposed cellular genes), and segmental duplications (duplicated genomic fragments). The large number of repetitive sequences involved during the process of evolution in plant genomes depending on their structure and mode of multiplications [13]. Moroever, long repeat sequences are spread throughout the chloroplast genomes of *Pinus* species. Recent studies have shown that most repeat sequences were positioned in the intergenic and intron regions whereas, limited repeat sequence were located in the coding regions of gymnosperm plastomes [1]. The diversity of the repeated sequences may provide valuable information for species adaptation to varying environmental condition.

In the present study, we will analyzed complete chloroplast genomes of or seventy-two *Pinus* species to identify structural variations and theircomparative genome analysis. We aimed toinvestugae comprehensive structural variations in *Pinus* genomes, examination of large repeat sequence variation in the plastid genome of *Pinus*, and reconstruction of phylogeny of major lineages of *Pinus* species based on complete chloroplast genome.

## Materials and methods

### Materials

The whole plastid genome dataset of seventy-two *Pinus* species and their three outgroups (*Picea glauca*, *Abies koreana* and *Abies nephrolepis*) were identified and downloaded from the NCBI (https://www.ncbi.nlm.nih.gov/). The *Pinus* complete cp genomes sequencing was annotated and further utilized for analysis.

### Chloroplast genome sequencing, annotation and divergence analysis

Data were used to generate a consensus sequence inside the software Geneious R v 8.0.2 (Biomatters Ltd., Auckland, New Zealand). Preliminary, the plastome annotation was turned using the program DOGMA (https://domainworld-services.uni-muenster.de/dogma/.). The stop and start codons are manually adjusted in Geneious R v 8.0.2. The round plastid genome map was drawn with the Organellar Genome DRAW v1.1 (OGDRAW) [14]. The sequence rearrangement of seventy-two plastomes was undertaken on Mauve Alignment [15]. To display interspecific variation, the alignments of the plastid DNA of the seventy-two genus *Pinus* were envisioned by mVISTA online software (https://genome.lbl.gov/vista/mvista/about.shtml) in the Shuffle-LAGAN mode and *P*. *squamata* specie was used as reference. The percentages of variable characters for non-coding and coding regions were counted via procedure given by Zhang et al. [16].

### Repeat sequence analysis

We found three types of repeats in complete chloroplast genome of seventy-two *Pinus* species: dispersed, tandem, and palindromicwhereas, web-based REPuter (https://bibiserv.cebitec.uni-bielefeld.de/reputer/) programmed was used to investigate these repeat sequences. The dispersed and palindromic repeats were used on following condition; (1) sequence identity 90%; (2) Hamming distance = 1 (3) repeat size minimum = 30 bp [17]. Tandem motifs (>10 bp in length) was identified using online software Tandem Repeats Finder (https://tandem.bu.edu/trf/trf.html) [18].

### Phylogenetic analysis

The complete dataset of *Pinus* genome sequence was aligned using MAFFT V 7.0.0 programmed [19]. Phylogenetic analysis was carried out using the cpDNA of all seventy two *Pinus* species (Table 1). These species were aligned with the Clustal W method of MEGA v7.0.18 software with manual inspection [20]. In addition, we included sequences from *Abies koreana*, *Abies nephrolepis* and *Picea gluca* as an outgroups. Maximum likelihood (ML) and maximum parsimony (MP) analysis were performed with the Akaike Information Criterion and an appropriate sequence evolution model selected by Model Test version 3.7. (AIC) [21]. Subsequently, one thousand (1000) bootstrap replicate was used to evaulate the support value of both ML and MP branches. PAUP* was used to calculate the phylogenetic reconstruction. Furthermore, the Bayesian phylogenetic analysis was operated using MrBayes v3.1.2 [22]. Markov Chain Monte Carlo (MCMC) was run over 3,000,000 generations, starting with an arbitrary tree and sampling topologies for every 100 generations. The first 2,500 trees (containing 25% of our samples) were burned (as recommended by MrBayes), and the remaining trees were used to build the 50% majorityrule consensus tree and estimate Bayesian posteriors of nodal support probabilities.

**Table 1:** The features of complete chloroplast genomes of seventy-two *Pinus* species.

Section	Species	Size (bp)	LSC (bp)	SSC (bp)	IR (bp)	Number of Protein Coding Genes	Number of rRNA Genes	Number of tRNA Genes	GC Contents (%)	Gene bank number
Double needle Section (Subgenera *Pinus*)										
	*P*. *jaliscana*	119,697	64,805	54,092	403	75	4	37	38.5	NC_035948
	*P*. *pringlei*	119,580	65,084	53,718	389	75	4	36	38.5	JN854189
	*P*. *lawsonii*	119,411	65,135	53,498	389	75	4	36	38.5	JN854188
	*P*.*oocarpa*	120,596	-	-	-	-	-	-	-	NC_035949
	*P*. *palustris*	119,149	65,190	53,181	389	75	4	36	38.5	JN854176
	*P*. *greggii*	119,480	64,849	53,853	389	74	4	36	38.5	NC_035947
	*P*. *patula*	119,356	65,130	53,448	389	75	4	36	38.5	JN854175
	*P*. *occidentalis*	119,826	65,204	53,844	389	75	4	36	38.5	JN854177
	*P*. *taeda*	120,534	65,610	54,146	389	75	4	36	38.5	NC_021440
	*P*. *pungens*	119,456	65,224	53,454	389	75	4	36	38.5	JN854167
	*P*. *caribaea*	119,528	64,924	53,634	399	75	4	36	38.5	JN854222
	*P*. *elliottii*	119,523	65,155	53,590	389	75	4	36	38.5	JN854202
	*P*. *glabra*	121,976	64,936	56,070	485	75	4	36	38.8	JN854199
	*P*. *muricata*	118,328	65,039	52,745	244	75	4	35	38.5	JN854180
	*P*. *radiata*	119,678	65,164	53,736	389	75	4	36	38.5	JN854165
	*P*. *coulteri*	119,785	65,141	53,866	389	75	4	36	38.5	JN854215
	*P*. *sabiniana*	118,929	64,830	53,129	485	75	4	36	38.5	JN854161
	*P*. *jeffreyi*	119,767	65,140	53,849	389	75	4	36	38.5	JN854193
	*P*. *engelmanii*	119,742	65,140	53,824	389	75	4	36	38.5	JN854201
	*P*.*douglasiana*	119,624	65,076	53,658	444	76	4	36	38.5	JN854205
	*P*. *arizonica*	119,965	64,899	54,084	492	75	4	37	36.4	JN854216
	*P*. *devoniana*	119,688	65,116	53,794	389	75	4	36	36.0	JN854208
	*P*. *montezeumae*	119,181	65,103	53,255	523	75	4	35	38.5	JN854183
	*P*. *hartweggii*	119,460	64,869	53,623	485	75	4	36	38.5	JN854206
	*P*.*pseudostrobus*	117,391	64,712	51,901	389	74	4	35	38.5	JN854178
	*P*. *clausa*	118,899	65,027	52,918	484	75	4	35	38.5	JN854217
	*P*. *roxburgii*	119,409	64,886	53,776	384	75	4	36	38.6	JN854162
	*P*. *pinea*	119,195	64,843	53,564	394	75	4	36	38.5	JN854173
	*P*. *heldrichii*	117,823	65,065	51,952	406	75	4	35	38.6	JN854195
	*P*. *halepensis*	118,947	64,750	53,237	394	75	4	36	38.5	JN854197
	*P*. *brutia*	120,570	64,990	54,610	485	75	4	36	38.5	JN854224
	*P*. *pinaster*	119,212	64,932	53,492	399	73	4	36	38.5	FJ899583
	*P*. *latteri*	119,279	65,069	53,432	389	75	4	36	38.6	JN854190
	*P*. *resinosa*	119,527	65,057	53,681	402	75	4	36	38.5	FJ899556
	*P*. *tropicalis*	118,924	65,002	53,133	389	75	4	36	38.5	JN854156
	*P*. *massoniana*	119,025	65,139	53,108	389	75	4	36	38.6	NC_021439
	*P*. *sylvestris*	115,909	64,415	50,661	420	75	4	37	38.6	KR476379
	*P*. *densiflora*	119,124	65,179	53,147	399	75	4	19	38.5	JN854210
	*P*. *fragilissima*	119,038	65,143	53,097	399	75	4	36	38.5	JN854200
	*P*. *kesiya*	118,986	65,179	53,009	399	75	4	36	38.6	JN854191
	*P*.*hwangshanensis*	118,993	65,175	53,020	399	75	4	36	38.5	JN854194
	*P*. *yunnanensis*	118,614	65,061	52,763	395	74	4	36	38.5	JN854151
Single needle Section (Subgenera *Strobus*)										
	*P*. *culminicola*	115,155	64,364	50,035	362	75	4	36	38.7	JN854213
	*P*. *discolor*	115,154	64,297	50,111	357	75	4	36	38.7	JN854207
	*P*. *cembroides*	115,919	64,394	50,581	460	75	4	36	38.6	JN854220
	*P*. *remota*	115,422	64,493	50,178	357	75	4	36	38.6	JN854164
	*P*. *quadrifolia*	115,508	64,385	50,367	362	75	4	36	38.7	JN854166
	*P*.*maximartinezii*	115,620	64,575	50,269	382	75	4	35	38.7	JN854184
	*P*. *rzedowskii*	115,934	64,652	50,508	380	75	4	36	38.6	FJ899557
	*P*. *nelsonii*	116,210	64604	50,845	367	74	4	35	38.7	EU998746
	*P*. *aristata*	116,918	64,251	51,707	480	75	4	35	38.7	FJ899567
	*P*. *bungeana*	116,751	64,311	51,490	475	75	4	36	38.8	NC_028421.
	*P*. *gerardiana*	116,668	64,296	51,339	516	75	4	36	38.7	EU998741
	*P*. *strobiformis*	116,200	64,230	51,108	474	75	4	36	38.7	JN854159
	*P*. *chiapensis*	116,197	64,524	50,895	392	75	4	36	38.8	JN854219
	*P*. *parviflora*	120,724	66,364	53,409	475	74	4	36	38.6	MG897304
	*P*. *wallichiana*	116814	-	-	-	-	-	-	-	JN854154
	*P*. *squamata*	117,327	64,706	51,825	398	74	4	36	38.7	MG897303
	*P*. *lambertiana*	116,958	64,604	51,592	379	75	4	35	38.8	EU998743
	*P*. *pumila*	114,087	64,553	48,762	384	75	4	36	38.7	JN854168
	*P*. *dalatensis*	116,657	64,533	51,321	393	75	4	36	38.8	JN854211
	*P*. *armandii*	116,998	64,337	51,711	389	75	4	36	37	NC_029847
	*P*. *morrisonicola*	116,636	64,104	51,770	381	74	4	36	38.7	MG897305
	*P*. *wangii*	118,073	65,598	51,521	476	74	4	36	38.7	MG897302
	*P*. *fenzeliana*	117,805	64,490	52,565	375	75	4	35	36.8	KX255674

## Results

### Genome features of seventy-two *Pinus* species

The complete chloroplast genomes of seventy-two *Pinus* species ranged in size from 114,087 (*P*. *pumila*) to 121,976 bp (*P*. *glabra*) (Table 1 and Fig 1). Plastid genomes had a quadripartite structure which present in most of the gymnosperm species. The complete genomes of *Pinus* species comprised of a large single copy (LSC) region ranged from 64,415 (*P*. *sylvestris*) to 65,610 bp *(P*. *taeda)*, and a small single copy (SSC) region ranged from 50,661 (*P*. *sylvestris*) to 56,070 bp (*P*. *glabra)*, and inverted repeats (IRs) ranged from 244 (*P*. *muricata*) to 492 bp (*P*. *arizonica*) in size (Table 1). The whole plastome of GC content was comparable to the *Pinus* species.

**Fig 1:** Gene map of 72 Pinus species. Genes drawn outside of the external circle are transcribed clockwise direction, and inside genes are transcribed clockwise directions. The Genes belong to varies functional group are colored coded. The darker gray region inside circle indicates GC content while the lighter gray color to AT content of the cp genome. Large single copy (LSC), small single copy (SSC), inverted repeat (IRs).

*Pinus* species complete cp genome consisted of 114 functional genes, with 36 tRNA, 4 rRNA and 74 protein-coding. Among 114 genes, 11 genes for small ribosome subunits, 9 genes for large ribosome subunits, 4 genes for DNA-dependent RNA polymerase subunits and 50 genes fragments were related to self-replication. The translational initiation factor (*infA*) gene, 38 genes for photosynthesis, 6 genes for ATP synthesis, and 11 genes encoding subunits of photosystem I (Table 2).

**Table 2:** Genes present in the seventy-two *Pinus* complete chloroplast genomes.

Gene group	Gene name				
Ribosomal RNA genes	*rrn16*	*rrn23*	*rrn5*	*rrn4*.*5*	
Transfer RNA genes	*trnI-CAU*	*trnL-UAA*	*trnI-GAU*	*trnL-UAG*	*trnL-CAA*
	*trnR-UCU*	*trnR-ACG*	*trnA-UGC*	*trnW-CCA*	*trnE–UUC*
	*trnV-GAC*	*trnV-UAC*	*trnT-UGU*	*trnF-GAA*	*trnT-GGU*
	*trnfM-CAU*	*trnP-UGG*	*trnG-GCC*	*trnP-GGG*	*trnS-GGA*
	*trnS-UGA*	*trnS-GCU*	*trnD-GUC*	*trnC-GCA*	*trnN-GUU*
	*trnE-UUC*	*trnY-GUA*	*trnQ-UUG*	*trnK-UUU*	*trnH-GUG*
	*trnG-GCC*	*trnM-CAU*			
Small Subunit of ribosome	*rps2*	*rps3*	*rps4*	*rps7*	*rps8*
	*rps11*	*rps12*	*rps14*	*rps15*	*rps18*
	*rps19*				
Large Subunit of ribosome	*rp12*	*rp114*	*rp116*	*rp120*	*rp122*
	*rp123*	*rp132*	*rp133*	*rp136*	
DNA-dependent RNA polymerase	*rpoA*	*rpoB*	*rpoC1*	*rpoC2*	
Translational initiation factor	*infA*				
Subunits of photosystem I	*psaA*	*psaB*	*psaC*	*psaI*	*psaJ*
	*psaM*	*ycf1*	*ycf2*	*ycf3*	*ycf4*
	*ycf10*				
Subunits of photosystem II	*psbA*	*psbB*	*psbC*	*psbD*	*psbE*
	*psbF*	*psbH*	*psbI*	*psbJ*	*psbL*
	*psbM*	*psbN*	*psbT*		
Subunits of cytochrome	*petA*	*petB*	*petD*	*petG*	*petL*
	*petN*				
Subunits of ATP synthase	*atpA*	*atpB*	*atpE*	*atpF*	*atpH*
	*atpI*				
Large subunit of Rubisco	*rbcL*				
Maturase	*matk*				
Protease	*clpP*				
Subunit of acetyl-CoA	*accD*				
C-type cytochrome synthesis gene	*ccsA*				

### Repeat sequence variations and genome structure comparison

In this study, we calculated three types of repetitions, i.e. dispersed, palindromic and tandem repeats. Among these repeat variations, a number of divisions and repeats were analyzed (S1 Table and Fig 2). We identified 5,943 repeats, among these repeats dispersed were most common with 2,612 (43.95%), followed by palindromic repeats with 1,921 (32.32%), and tandem repeats with 1,410 (23.72%) (Fig 1). Majority of repeats found circulated in intergenic regions and few were situated within generic regions. *P*. *nelsonii* were the most dispersed repeated sequences (76) followed by *P*. *pseudostrobus* (63) palindromic repeats whereas, *P*. *sabiniana* showed lowest number tandem repeats with only (13) tandem repeats (S1 Table).

**Fig 2:** A histogram of the number of repeats found in the seventy-two Pinus chloroplast genomes. (a) The number of repeats in subgenus Pinus (b) Number of repeats in subgenus Strobus.

For sequence identity analysis mVISTA was used with *P*.*squa*mata sequence as reference (S1 Fig). It was observed that 72 *Pinus* species hold large number of sequence similarity however, lesser degree of variation was also observed. It is worthy to mention that non-coding regions displayed high levels of divergence compared to coding regions. The outcome helped to identified hotspot divergent regions on *Pinus* cp genome (S1 Fig). The non-coding regions displayed sequence divergence, and percentage of variation ranged from 0 to 13.78% with an average of 4.96%, whereas, the percentage variation in coding region ranged from 0 to 9.98% with an average of 2.54% (Fig 3). Furthermore, we discovered that IR region has a lower number of mutations and is highly conserved in *Pinus* species. It noteworthy, we identified seven genes(*trnD-GUC*, *trnY-GUA*, *trnH-GUG*, *ycf1*, *trnL-CAA*, and *trnV-GAC*) at LSC and SSC region located within the non-coding regions showing greater levels of variation, with ability to act as divergence hotspot regions.

**Fig 3:** Variable characters percentage in homologous regions of Seventy-two Pinus species of chloroplast genome (a) Coding region (b) Non coding region. The homologous regions are oriented according to their locations in the chloroplast genome.

### Phylogenetic relationships of *Pinus* species

The 72 *Pinus* chloroplast genome sequences were used for phylogenetic analysis. Under the GTR+G+I model, we re-constructed three independent phylogenetic trees through different analytical methods: maximum parsimony (MP), maximum likelihood (ML), and Bayesian inference (BI) (Fig 4). Among investigated species, the phylogenetic analysis displayed congruent topologies, although the bootstrap value was kept slighlty different for all phylogenetic trees. The phylogenetic tree further divided into two clades, single-needle section (subgenus *Strobus)* and double-needle section (subgenus *Pinus* species) (Fig 4). We found that *P*. *wangii*, *P*. *fenzeliana*, *P*. *morrisonicola* and *P*. *armandii* posses close relationships and catageorized in the single needle section. In addition, the *P*. *parviflora*, *P*. *chiapensis* and *P*. *wallichiana* were closely related to subgenus *Pinus*.

**Fig 4:** Phylogenetic tree obtained from whole cp genome (A) The numbers above the branches represent bootstrap values greater than 50% for ML (left) and MP (middle) analyses, and Bayesian posterior probabilities (right). A dash shows a bootstrap value less than 50%.

## Discussion

### Features of cp genomes of *Pinus* species

The chloroplast genome of higher plants is circular molecule with a length of 120–160 kb with approximately 130 genes [23]. The structure and organization of thes genes found similar among the 72 *Pinus* species under investigation. Moreover, similar GC level for 72 *Pinus* species was observed which is less common for most of the terrestrial plants [23]. IRs contraction and expansion are extensively exhibited in many lands plant species. The, large IRs played a significant role in maintaining the constancy of whole plastome [24]. Small IR region may cause variations in genome structure and content of plastome [25]. Interestingly, in present study, we detected small IR regions in all investigated *Pinus* species (244 to 492 bp). Following results displayed that in certain genes have variations for structure and contents compared to whole cp genome of *Pinus* species [26].

previous investigations has exhibited that repeat sequences have performed significant roles in genome re-organization and recombination [27]. Among 72 *Pinus* species *P*. *nelsonii* genome had large numbers of repeats (76), whereas, *P*. *pseudostrobus* genome have (63) repeats. In contrary, *P*. *sabiniana* displayed lowest number of (13) repeats (S1 Table and Fig 2). However, the tandem, dispersed, and palindromic repeats distributions were comparable for all *Pinus* species. A large number of repeats could maintain cp genomes constants, similar results reported by Zhang et al [16]. The repeat sequence displayed similar genes function rearrangement for further study in population genetics and *Pinus* species evolution [2].

### Comparative analysis of the genomic structure

The complete chloroplast genome of *Pinus* species displayed a very low genetic divergence. Sequence alignment of 72 plastids genomes were compared, and used for sequence identity analysis via mVISTA programe, keeping *P*. *squamata* as a reference specie (S1 Fig). The similarity analysis exhibited a high sequence comparison across the plastid genomes having sequence identities below 90%. However, a low divergence region identified in LSC and less mutation rate in IRs region. In addition, the divergent hotspot regions (*trnD-GUC*, *trnY-GUA*, *trnH-GUG*, *ycf1*, *trnL-CAA*, *trnK-UUU and trnV-GAC*) were found in non-coding regions of some tRNA sequences. Several repetitive sequences were equally distributed in the divergence hotspot regions. These hotspot regions can be utilized for phylogenetic study and provide DNA barcoding for future evolutionary studies of gymnosperm species [28].

### Phylogenetic relationships of *Pinus* species

The whole plastome phylogenetic analysis has been commonly undertaken in land plants [29]. During recent decade, a study has revealed phylogenetic relationship and comparisons of numerous protein-coding genes present in the chloroplast genomes [30]. That improved our understanding for phylogenetic relationship and molecular studies among *Pinus* species [31].

The current study used phylogenetic analysis based on entire cp genome sequence of 72 *Pinus* specieshaving *P*. *glauca*, *A*. *nephrolepis*, and A. koreana serving as outgroups. Using ML, MP, and BI methods, we created a concurrent phylogenetic tree with a wide range of supported values (Fig 4). The phylogenetic tree of *Pinus* species was divided into two groups that corresponded to single needle sections and double needle sections. Among these sequenced species, single-needle section species i.e., *P*. *morrisonicola* and *P*. *wangii* catagorized in the same clade, showing a close relationship with each other. Moreover, these two species showed a high similarity in their chloroplast genome sequences [31]. In addition, the phylogenetic tree revealed *P*. *bungeana* and *P*. *gerardiana* has a close relationship with each other [32]. The phylogenetic results exhibited *P*. *clausa* showed a sister clade to the *Pinus* species [33].

## Conclusion

The present study determined the whole chloroplast genome a rich source to understanf the evolutionary history. The cp genomes of *Pinus* species, genome structure and order were similar in nature. Moreover, the location and distribution of repeat sequences were determined, and common pairwise sequence divergences among cp genomes of interrelated species were identified. The whole genome sequencing proved to be a significant knowledge for plant taxonomic positioning. The main findings based on complete chloroplast genome of *Pinus* species divided into two sections, single needle sections and double-needle sections of *Pinus* species. The phylogenetic relationships dependent on the cp genome greatly developed our understanding on phylogeny of *Pinus* species. Comparative analyses of plastid genome sequences provide DNA markers for easy identification and classification. These results will provide supportable confirmations and prove a solid basis for the improvement of chloroplast genome in *Pinus* species.

## Supporting information

S1 Fig Sequence alignment of chloroplast genomes of Pinus species. mVISTA-based identity plots viewing identity between seventy-two Pinus species cp genomes. The vertical scale indicates the percentage identity, ranging from 50% to 100%. Divergent hotspot refers to the places with more variable sites compared to another region.
(DOCX)

S1 Table Repeat sequences analysis in seventy-two Pinus species based on complete chloroplast. (DOCX)
